The article "miR-874 inhibits gastric cancer cell proliferation by targeting SPAG9" was retracted in 2025. Reasons: manipulated images; plagiarized images; duplicated images; overlap with other authors' work.

# *miR****-****874* inhibits gastric cancer cell proliferation by targeting *SPAG9*

**DOI:** 10.1186/s12885-020-06994-z

**Published:** 2020-06-05

**Authors:** Qin Hui Sun, Zong Xiu Yin, Zhi Li, Shu Bo Tian, Hong Chang Wang, Fang Xu Zhang, Le Ping Li, Chun Ning Zheng, Shuai Kong

**Affiliations:** 1 Department of Gastrointestinal Surgery, Shandong Provincial Hospital, Cheeloo College of Medicine, Shandong University, Jinan, 250021 China; 2 Department of Respiration Medicine, Jinan Central Hospital Affiliated to Shandong University, Jinan, 250013 China; 3 Department of Operating Room, Jinan Central Hospital Affiliated to Shandong University, Jinan, 250013 China; 4 Department of Gastrointestinal Surgery, Shandong Provincial Hospital Affiliated to Shandong First Medical University, Jingwu Road No.324, Jinan, 250021 China; 5 School of Clinical Medicine, Weifang Medical University, Weifang, 261042 China

**Keywords:** Gastric cancer, miR-874, SPAG9, Proliferation, Apoptosis

## Abstract

**Background:**

microRNAs (miRNAs) play essential roles in the development and progression of gastric cancer (GC). Although aberrant *miR-874* expression has been reported in various human cancers, its role in GC remains obscure.

**Methods:**

*miR-874* expression was assessed by real-time quantitative polymerase chain reaction (RT-qPCR) in 62 matched GC and adjacent normal tissues, as well as in GC cell lines and immortalized human gastric epithelial cells. CCK8 assay, colony formation assay, and flow cytometry were used to assess the role of miR-874 in GC cell proliferation and apoptosis in vitro. Additionally, to determine the effects of *miR-874* on GC cell proliferation and apoptosis in vivo, BALB/c nude mice were injected with GC cells transfected with a *miR-874* mimic. The role of *miR-874* in *SPAG9* expression was assessed by luciferase assay, Western blotting, and RT-qPCR.

**Results:**

*miR-874* was downregulated in GC cell lines and tissues. *miR-874* overexpression in GC cells led to inhibition of cell proliferation and induction of apoptosis. Moreover, *SPAG9* was identified as a direct *miR-874* target, the expression of which was suppressed by *miR-874*. *SPAG9* overexpression markedly promoted GC cell proliferation.

**Conclusions:**

*miR-874* inhibited cell proliferation and induced apoptosis in GC cells. *SPAG9* downregulation was crucial for the tumor-suppressive effects of *miR-874*. Hence, the *miR-874*/*SPAG9* axis could serve as a novel therapeutic target in GC.

## Background

Gastric cancer (GC) is a common malignancy and important cause of mortality and morbidity, both in China and worldwide [1]. The 5-year survival rate of patients with GC after radical surgery ranges from 30 to 50%; the high malignancy and heterogeneity of GC, as well as its poor differentiation, are primary causes of poor prognosis [2]. Despite advances in surgical interventions, chemotherapy, targeted therapies, and immunotherapy, the overall prognosis of GC remains poor [3]. Therefore, elucidation of molecular mechanisms underlying GC cell proliferation, survival, and metastasis are imperative for developing novel therapeutic interventions GC. Additionally, identification of robust prognostic biomarkers and GC classification based on molecular profiles would enable personalized treatment of GC.

MicroRNAs (miRNAs) are 21–25-nucleotide, single-stranded, non-coding RNAs. miRNAs specifically bind to the 3′ untranslated region (3′-UTR) of target genes, which facilitates mRNA degradation or translation suppression. It has become evident that miRNAs play crucial roles in various biological processes, such that they regulate the expression of approximately 30% of all mRNAs expressed in a cell. Additionally, numerous miRNAs have been implicated in various human cancers, exerting either tumor suppressor or oncogenic functions [4]. *miR-105* [5], *miR-664a-3p* [6], *miR-451a* [7], and *miR-18b* [8] have recently been identified as oncogenes in GC; moreover, *miR-223-3p* [9], *miR-99b-3p* [10], and *miR-1297* [11] have been shown to suppress GC development and progression. *miR-874* is a newly identified miRNA, which plays key roles in various malignancies, including nasopharyngeal carcinoma [12], non-small cell lung cancer [13], colorectal cancer [14], and hepatocellular carcinoma [15]. However, the role of *miRNA-874* in GC remains unclear.

The oncogene sperm-associated antigen 9 (SPAG9) is a member of the cancer/testis antigen family; its expression is regulated by various miRNAs, including *miR-524* [16] and *miR-200a-3p* [17]. In this study, we investigated the relevance of *miR-874* in GC development and progression, by assessing the effects of *miR-874* on GC cell proliferation, as well as the relationship between *miR-874* and *SPAG9*.

## Methods

### Patients and ethics

Sixty two patients (35–72 years old) including 49 males and 13 females with surgical tumor specimens and adjacent non-tumor tissues were collected from Shandong Provincial Hospital Affiliated to Shandong First Medical University (Jinan, Shandong) after receiving written informed consent during July 2017 to May 2018. The histological diagnosis was made on sections stained with hematoxylin and eosin, according to the World Health Organization (WHO) classification guidelines. None of our study patients had received preoperative chemotherapy or radiotherapy. The study was approved by the Human Ethics Committee of Shandong Provincial Hospital Affiliated to Shandong First Medical University.

### Cell culture and transfection

Human gastric mucosal epithelial cells (GES-1), human GC cell lines (MKN-74, BGC-823, MGC-803, MKN-45) in this study were purchased from Cell Bank of Chinese Academy of Sciences (Shanghai, China) and used in our experiments. Cells were cultured into T25 flasks in RPMI-1640 medium supplemented with 10% FBS, and grown in a humidified chamber supplemented with at 37 °C with 5% CO_2_. The *miR-874* mimic and inhibitor, *SPAG9* siRNA (si-SPAG9) and *SPAG9* were obtained from Santa Cruz. Transfection was achieved using the LipofectamineTM 3000 kit (Invitrogen) according to the manufacturer’s instructions.

#### Real-time quantitative polymerase chain reaction (RT-qPCR)

Total RNA was extracted from tissues or cultured cells with TRIzol reagent (Thermo Fisher Scientific) according to the protocol [18]. RT-qPCR was performed using SYBR Green PCR master mix (Applied Biosystems) in a total volume of 20 μl on 7900HT Fast Real-Time PCR System (Applied Biosystems) as follows: 95 °C for 30 s, 40 cycles of 95 °C for 5 s, and 60 °C for 30 s. A dissociation step was performed to generate a melting curve to confirm the specificity of the amplification. The U6 small nuclear RNA and GAPDH mRNA were used to normalize the expression for *miR-874* and *SPAG9* mRNA, respectively. The following primers were as follows: *SPAG9* forward primer: 5′-CAA GGC GGA TCT AAA GCT ACC − 3′, reverse primer: 5′-TTG GCG CAT CTG TAA CCT TCA-3′, *GAPDH* forward primer: 5′- CTG GGC TAC ACT GAG CAC C − 3′, reverse primer: 5′- AAG TGG TCG TTG AGG GCA ATG-3′, *U6* small nuclear RNA forward primer: 5′-CTC GCT TCG GCA GCA CA − 3′, reverse primer: 5′-AAC GCT TCA CGA ATT TGC GT-3′; *miR-874* forward primer: 5′-CAC GCA CCA GGG TAA GAG AG-3′, reverse primer: 5′-CCA GCC AGT CGG TCC CT-3′.

### Luciferase activity assay

According to TargetScan (http://www.targetscan.org) and MiRanda (http://www.microrna.org/microrna/home.do) databases, the wild-type SPAG9 3’UTR (SPAG9-Wt) or the mutant SPAG9 3’UTR (SPAG9-Mut) was constructed into the pGL3 luciferase reporter vector. The above luciferase reporter plasmid was co-transfected with miR-874 mimic or NC mimic into BGC-823 cells, and the pRL-TK luciferase reporter vector was used as negative control. Luciferase assay was performed the firefly luciferase 48 h post-transfection and measured using the Dual-Luciferase® Reporter Assay System (E1910, Promega Corporation, Madison, WI, USA).

### Cell proliferation assay

CCK8 assay in this study was performed to determine the cell proliferation. In brief, cells were added into 96-well plates and cultured for another 48 h. Then 20 μl 5 mg ml^− 1^ CCK-8 solution was added for another 4-h culture. With the supernatant removal, 150 μl dimethyl sulfoxide was added into each well of the plate in a shaking table at low speed at room temperature for 10 min. The optical density (OD) at 450 nm was measured.

### Colony formation assay

The capacity of cell proliferation was further detected using the colony formation assays. In brief, after cultured for 14 days, transfected BGC-823 cells (~ 3 × 10^4^/6-well plate) were fixed with formaldehyde (4%) and then stained with 0.5% crystal violet solution. Lastly, a light microscope was used to count the number of colonies (> 50 cells).

### Cell apoptosis analysis

BGC-823 cells were collected, washed twice with cold 1 × PBS. Then the cells were binding buffer to a concentration of 1–5 × 10^6^/ml. Next, 100 μl of cell suspension was added into a 5 ml tube followed by adding 5 μl of Annexin V/FITC and 5 μl of Propidium Iodide (PI) into the tube. After being incubated for 15 min in the dark, 400 μl of 1 × Annexin V binding buffer were added into the tube. The cells were analyzed by flow cytometry (BD, USA).

### Western blot analysis

The total protein content was isolated from collected cell samples using radioimmuno-precipitation assay (RIPA) buffer (Thermo Fisher Scientific, Waltham, MA) on ice for 30 min and centrifuged at 10000 g for 30 min. Subsequently, the protein concentration in each sample was measured by utilizing a BCA assay (Thermo Fisher Scientific, Waltham, MA), the pallets were discarded and supernatants were mixed with the loading buffer for electrophoresis. Proteins were separated by electrophoresis on 10% SDS-polyacrylamidegels, before being transferred to polyvinylidene difluoride membranes (MerckMillipore, Billerica, MA, USA). Blots were blocked with a 5% skim milk solution and incubated overnight with an antibody against SPAG9 (1:1000; Abcam, UK) or GAPDH (1:5000, Santa Cruz Biotechnology, USA). Membranes were then exposed to the corresponding horseradish peroxidase-conjugated secondary antibodies for 2 h at room temperature. Bio-Rad CheciDOC XRS chemiluminescence imaging system was performed to detect the bands, and the luminescence images were acquired for quantitative analysis.

### In vivo tumor growth model

All mouse experiments were approved by the Ethics Committee of the Shandong Provincial Hospital Affiliated to Shandong First Medical University. BALB/c nude mice (female, 4–6 weeks) were randomly divided into NC group, *miR-874* mimic group and *miR-874* inhibitor group (*n* = 6 per group). The cells of each group were collected and made into single-cell suspension with a concentration of 5 × 10^6^ cells/mL. The mice were sacrificed by cervical dislocation at the end of 4 weeks, and all the solid tumors were stained with TUNEL staining to observe the apoptosis of the tumor.

### Statistical analysis

All data were presented as mean ± standard deviation (SD) and analyzed using a professional SPSS software 20.0 (SPSS Inc., Chicago, UL, USA). Differences between two groups were analyzed using student’s t-test and among three or more groups were analyzed by one-way ANOVA. *P* < 0.05 was considered statistically significant.

## Results

### *miR-874* is downregulated in GC

*miR-874* expression levels in 62 matched GC and tumor-adjacent normal tissues were measured with RT-qPCR. Notably, *miR-874* was expressed at substantially lower levels in GC tissues, compared to paired normal tissues (Fig. 1a). Similarly, *miR-874* was expressed at considerably lower levels in GC cell lines MKN-74, BGC-823, MGC-803, and MKN-45, compared to GES-1 cells (Fig. 1b); BGC-823 cells exhibited the lowest *miR-874* expression.

**Fig. 1:** Down-regulation of miR-874 was observed in GC. The expression of miR-874 was detected via RT-qPCR in GC tissues (**a**). The expression of miR-874 was detected in MKN-74, BGC-823, MGC-803, MKN-45 and GES-1 cells (control) (**b**). ** *P* < 0.01. GC, gastric cancer; RT-qPCR, reverse transcription-quantitative PCR

### *miR-874* inhibits proliferation and promotes apoptosis in vitro in GC cells

Various GC cell lines were transfected with a *miR-874* mimic, and *miR-874* overexpression was confirmed by RT-qPCR (Fig. 2a). Subsequently, the proliferation rate of GC cells was measured using the CCK8 method and colony formation assays. Both assays revealed that *miR-874* overexpression dramatically suppressed cell proliferation in all three GC cell lines (Fig. 2b, c). The role of *miR-874* in cell apoptosis was also evaluated by flow cytometry; the *miR-874* mimic significantly increased GC cell apoptosis, compared with the control group (Fig. 2d).

**Fig. 2:** miR-874 inhibited cell proliferation and promotes cell apoptosis in vitro in GC. RT-qPCR was performed to detect the miR-874 expression in BGC-823, MKN-74 and MGC-803 cells contained miR-874 mimics or inhibitor (**a**). CCK8 (**b**) and colony formation (**c**) assay was performed to detect the proliferation of cells containing miR-874 mimics or inhibitor. The cell apoptosis was measured in cells containing miR-874 mimics or inhibitor via flow cytometer (**d**). * *P* < 0.05; ** *P* < 0.01. GC, gastric cancer; RT-qPCR, reverse transcription-quantitative PCR

### *miR-874* inhibits proliferation and promotes apoptosis in vivo in GC cells

To further confirm the tumor-suppressive effect *of miR-874*, BALB/c GC xenograft models were employed. Notably, *miR-874*-overexpressing tumors were significantly smaller at 4 weeks after cancer cell implantation, compared to control tumors (Fig. 3). Conversely, *miR-874* inhibition accelerated tumor growth in our GC mouse model. Furthermore, TUNEL assay analysis revealed enhanced cancer cell apoptosis in *miR-874*-overexpressing tumors.

**Fig. 3:** miR-874 inhibited cell proliferation and promoted cell apoptosis in vivo in GC*.* Tumor size (**a**), tumor volume (**b**) and tumor weight (**c**) of mice were measured. TUNEL assay was detected the apoptosis in the tumor tissues (**d**). * *P* < 0.05; **P < 0.01

### *miR-874* directly targets *SPAG9* in GC cells

Using miRNA seed sequence targeting prediction analysis, a potential *miR-874* binding site was identified in the 3’UTR of *SPAG9* (Fig. 4a). Subsequent use of a dual-luciferase reporter assay system showed that luciferase activity was significantly reduced in pGL3-PIK3CA-SPAG9-expressing cells after transfection with the *miR-874* mimic, compared with pGL3-PIK3CA-NC and pGL3-PIK3CA-SPAG9-Mut cells (*P* < 0.01); this finding confirmed that *miR-874* binds to the 3’UTR of *SPAG9*, thereby suppressing its expression (Fig. 4b). RT-qPCR and Western blotting were also performed to confirm the effects of *miR-874* on SPAG9 expression at the mRNA and protein levels, respectively. Notably, transfection with the *miR-874* mimic significantly reduced SPAG9 protein levels (*P* < 0.01). Conversely, *miR-874* inhibition increased SPAG9 protein levels (*P* < 0.001) (Fig. 4c). Consistent with these findings, RT-qPCR analysis showed that the mRNA levels of *SPAG9* were significantly reduced after transfection with the *miR-874* mimic (Fig. 4d). Overall, these results suggest that *miR-874* directly binds *SPAG9*, thus suppressing its expression.

**Fig. 4:** miR-874 directly targeted SPAG9 in GC cells. The binding site of miR-874 on the 3′-UTR of SPAG9 (**a**). Luciferase activity of MCG-823 cells transfected with miR-874 mimics in the presence of pGL3-PIK3CA-SPAG9 Wt or pGL3-PIK3CA-SPAG9 Mut was detected (**b**). Western blot (**c**) and RT-qPCR (**d**) were performed to detect the effect of miR-874 on SPAG9 both at protein level (full-length blots are presented in Additional file 1) and mRNA. ** *P* < 0.01. GC, gastric cancer

### *miR-874* regulates the progression of GC by modifying *SPAG9* expression

BGC-823 cells were transfected with *SPAG9*, *miR-874*, or a combination of these (Fig. 5a). Importantly, *SPAG9* overexpression significantly promoted cell proliferation (Fig. 5b, c), whereas it inhibited cell apoptosis (Fig. 5d). Transfection with the *miR-874* mimic reversed the effects of *SPAG9* overexpression on GC cell proliferation and apoptosis.

**Fig. 5:** miR-874 regulated the progression of GC through affecting SPAG9 expression. The mRNA expression of SPAG9 was measured in cells containing SPAG9 plasmid with or without miR-874 (**a**). The cell proliferation in cells containing SPAG9 plasmid with or without miR-874 via CCK8 (B) and colony formation assay (**c**). The cell apoptosis was measured in cells containing SPAG9 plasmid with or without miR-874 via flow cytometer (**d**). *P < 0.05, **P < 0.01. GC, gastric cancer

## Discussion

GC incidence and mortality remain high [19]. With recent advances in the fields of molecular and cell biology, the understanding of molecular mechanisms underlying cancer has advanced considerably. Additionally, many genes have been shown to regulate cancer cell proliferation [20]. Notably, gene therapy has emerged as a promising therapeutic approach for cancer, as well as for other human diseases. Several miRNAs have been shown to regulate cell differentiation, proliferation, and survival, through binding interactions with complementary target mRNAs [21]. *miR-874* has recently been identified as a tumor-suppressor and is often downregulated in certain types of cancer, including GC [22]. In this study, we confirmed that *miR-874* expression was reduced in GC tissues and cells. We also demonstrated that *miR-874* overexpression suppressed GC cell proliferation and promoted apoptosis.

Furthermore, we investigated the mechanism underlying the tumor-suppressive effects of *miR-874* in GC. Aberrant *SPAG9* expression has been reported in several malignancies, including renal, breast, thyroid, and cervical cancer. However, the relevance of *SPAG9* in human GC remains elusive. In the present study, we identified *SPAG9* as a *miR-874* target. We also demonstrated that *SPAG9* overexpression enhanced cell proliferation and inhibited cell apoptosis in GC cells. Consistent with these findings, a recent study showed that *SPAG9* overexpression promoted proliferation in human prostate cancer cells [23]. Furthermore, *SPAG9* has been shown to regulate HEF1 expression, promoting epithelial to mesenchymal transition in urothelial carcinoma in a Rac1 pathway-dependent manner [24]. In prostate cancer, *SPAG9* promotes cell survival, angiogenesis, and tumor metastasis by activating the MAPK signaling pathway [25].

## Conclusions

In conclusion, we demonstrated that *miR-874* inhibited cell proliferation and induced apoptosis in GC cells. We also identified the *SPAG9* oncogene as a target of *miR-874* and showed that *SPAG9* downregulation was crucial for the tumor-suppressive effects of *miR-874*. Therefore, the *miR-874*/SPAG9 axis could serve as a novel therapeutic approach for GC.

## Supplementary information

**Additional file 1.** Original data of western blot (SPAG9 and GAPDH) in Fig. 4, the cropping of the blot by figure processing software was clearly mentioned with red rectangle.

## Data Availability

All data generated or analysed during this study are included in this published article and its supplementary information files.

## Abbreviations

miRNAs: microRNAs
GC: Gastric cancer
SPAG9: Sperm associated antigen 9
CT: Cancer testis
RIPA: Radioimmuno-precipitation assay
ANOVA: Analysis of variance
3’UTR: 3′-Untranslated region
